# The Value of CT 3D Reconstruction in the Classification and Nursing Effect Evaluation of Ankle Fracture

**DOI:** 10.1155/2021/9596518

**Published:** 2021-08-09

**Authors:** Pan Xue, Xue Chen, Si Chen, Yuanyuan Shi

**Affiliations:** ^1^Department of Orthopedics, The Second Hospital of Jilin University, Changchun 130041, China; ^2^Geriatric Medicine, The Second Hospital of Jilin University, Changchun 130041, China; ^3^Department of Nursing, The Second Hospital of Jilin University, Changchun 130041, China

## Abstract

**Aim:**

To study the application value of ankle fracture classification and diagnosis. In this paper, the clinical data of 100 cases of ankle fracture patients admitted from May 2020 to May 2021 were analyzed by CT 3D reconstruction. All patients received surgical treatment and underwent spiral CT 3D reconstruction and X-ray examination before surgery. The results showed that 20 cases (20.00%) of the 100 cases were PER, 24 cases (24%) of the 100 cases were PAB, 31 cases (31%) of the 100 cases were SER, and 25 cases (25%) of the 100 cases were SAB, respectively.

**Conclusion:**

The diagnostic accuracy of CT 3D reconstruction for different types of ankle fracture is higher than that of X-ray, and the differences are statistically significant (*P* < 0.05). CT 3D reconstruction is applied in the early diagnosis of ankle fracture, which can accurately detect the classification of patients. It has important clinical application value and can be used as the first choice for the early classification diagnosis of ankle fracture.

## 1. Introduction

Manic joint fracture is the most common intra-articular fracture, accounting for about 3.9% of systemic fractures, which is most likely to occur in young adults. Due to the different mechanism of injury, the manifestation of ankle fracture is different. With the in-depth understanding of the anatomy, function, biomechanical properties of the disc joint, and injury mechanism, the classification methods pay more attention to comprehensive factors, such as the location of foot injury, the magnitude and direction of external force, the relationship between inlay and fracture, and the process and degree of fracture [1]. The area of ankle joint is smaller than that of hip joint and knee joint, but the pressure is the largest among the three. In addition, the ankle joint is close to the ground, and the load-bearing stress acting on it cannot be buffered. Therefore, the treatment of ankle fracture is higher than that of other parts. The importance of anatomical reduction of ankle joint has become a consensus. Uneven articular surfaces or poor reduction of the ankle after a manic joint fracture can lead to limited joint movement, pain, and traumatic arthritis. How to choose the most appropriate treatment is closely related to the classification and diagnosis of fracture. Currently, there are three commonly accepted and commonly used classifications in clinical practice: mechanical classification, surgical classification, and Ashurst–Bromer classification. The above classification methods have their own advantages, but for disc fracture, there are many factors that affect the prognosis, and there is no effective and comprehensive classification method to judge the prognosis at present. In addition, the classification diagnosis mentioned above is usually based on radiography, but due to the special anatomical structure of foot manic part, conventional ankle radiographs are difficult to comprehensively and clearly show the X-ray and bone fragments, which makes the classification diagnosis of ankle more difficult [2]. In recent years, with the continuous progress and improvement of spiral CT three-dimensional reconstruction technology, fracture positioning is more accurate and intuitive and can better display the spatial morphology of ankle fracture, which provides convenience for classification and diagnosis.

Injures of the primary triangle of the ankle joint can be divided into acute and chronic injuries. The acute injury is usually manifested by tenderness and hematoma of the angular band at the medial malleolus, while the chronic injury is manifested by dull pain of the medial sulcus of the ankle joint, which is typically caused by palpation of the anterior medial malleolus. There is obvious tenderness before and below the tip of the medial malleolus, subcutaneous spots can be seen, and there is a sense of depression or emptiness when pressing the inner side of the heel joint. Due to acute injury, patients have obvious clinical symptoms, so they can usually attract the attention of patients and take corresponding measures to prevent the aggravation of ligament damage. However, chronic injury is not easy to attract the attention of patients because the symptoms occur from time to time. As a result, the triangular ligament cannot rest, but it is more likely to lead to the instability of the medial disc joint, which is mainly manifested as “hitting the soft leg” when walking on uneven ground, downhill, or down stairs [3]. Qi Xiaoyang et al. pointed out that the smoothness and displacement of the ankle joint surface are closely related to the elasticity of the joint ligament and the articular surface stress. If the articular surface shifts outward by 1 mm, the contact area of the tibial talar joint will be reduced by about 40%. If the displacement or shortening of the articular surface is more than 2 mm or external rotation is more than 5°, the stress of the ankle will be abnormally distributed, which is very easy to lead to many complications such as traumatic arthritis. Therefore, in case of ankle fracture, patients should be classified and diagnosed in time in the early stage, so that clinicians can design a reasonable surgical treatment plan to ensure the postoperative rehabilitation of patients and achieve the purpose of effective anatomical reduction and internal fixation [4]. In the past, the diagnosis of ankle fractures mostly relied on conventional CT plane scan and X-ray film. However, the use of X-ray film is easy to appear like the overlapping image of ankle fractures and unable to clearly show the small broken end displacement, fracture line, articular surface, and other conditions, resulting in a high rate of missed diagnosis and misdiagnosis. Two-dimensional CT has a higher resolution than X-ray film without overlapping images, but due to the poor stereoscopic sense of the sectional plane images, it is unable to comprehensively and accurately evaluate the overall situation of ankle fracture, and its application also has certain limitations [5].

Hinb et al. proposed the “foot free suspension test” to check whether the triangle facing belt is damaged. The specific methods are as follows: the examinee holds the subject's heel on the affected side with one hand and the ipsilateral cavity bone with the other hand and imposes a valgus force and valgus force on the heel, respectively. The degree of valgus is checked and then compared with the contralateral side, so as to infer the damage of the triangular zone. In addition, the drawer test commonly used in orthopedics to check the degree of relaxation of Bremsstrahlung can also be used to infer the condition of sonic injury of the primary triangular band. The principle of treatment of manic joint fracture is to completely remove the intra-articular bone fragments and achieve anatomic reduction at the ankle point. However, it has been reported abroad that it is very difficult to completely rely on surgical anatomical reduction for the treatment of ankle fractures, and it is almost impossible to achieve anatomical reduction by surgical treatment, not because of the limited surgical techniques, but because of the failure to correctly evaluate the degree of fracture injury of patients before surgery [6]. So, an accurate assessment of preoperative plan formulation, treatment effect of surgery, has important meaning, and 3D reconstruction technology in this advantage is particularly prominent in the presence of displaced fractures, more blocks, more severe compression or comminuted fracture, intra-articular fractures cases, which ordinary methods do not have. Through clinical practice, many scholars at home and abroad put forward that 3D reconstruction can not only display the trend of fracture line, the damage of joint surface, joint cavity and joint capsule, the position of fracture fragments, dislocation, and subluxation comprehensively, intuitively, three-dimensional, and accurately but also can accurately display the subtle anatomical structure of ankle joint and clearly show the bleeding of soft tissue around manic joint. It is not only conducive to judge the fracture classification and provide more effective and valuable information but also has far more advantages than the traditional examination methods. Clinical practice also shows that preoperative preparation can be fully completed through three-dimensional reconstruction examination and further evaluation of the risk of surgery, so as to achieve anatomical reduction of fracture as far as possible and maximize the recovery of patients' manic joint function [7].

The innovation of this paper: spiral CT reconstruction is targeted at different fracture sites of patients and can comprehensively display the specific situation of ankle fracture, which can not only eliminate image overlap but also improve the accuracy of classification diagnosis of ankle fracture and provide reliable diagnostic basis for patients' future treatment.

## 2. Materials and Methods

### 2.1. General Information

Retrospective analysis was performed on the imaging and clinical data of 100 patients with ankle joint fracture admitted to the hospital of the author from May 2020 to May 2021. This study was approved by the medical ethics committee of the hospital of the author. Among the 100 patients, 59 were male and 41 were female. The average age was (44.79 ± 10.51) years from 21 to 67 years old.

### 2.2. Inclusion Criteria

Inclusion criteria: (1) all patients had new ankle fractures; (2) no pathological fracture was found; (3) daily life before fracture can be self-care; (4) have good language skills; (5) all patients received surgical treatment; (6) complete clinical data. Exclusion criteria: (1) patients with severe consciousness impairment, cognitive impairment, and mental disorder; (2) patients with systemic blood diseases; (3) patients with combined diseases that have influence on imaging examination.

## 3. Methods

All patients underwent X-ray examination and spiral CT three-dimensional reconstruction.

1. Data collection preoperative imaging examination data, physical sign examination data, trauma history, and intraoperative conditions of the patients were collected, and relevant imaging images were analyzed using Digimizer measurement software. Anteroposterior radiographs of the ankle included TFCS, TFO, coin sign, and Shenton line. Ankle acupoint films: tibial talus angle, talus leg and foot, talus tibial space (TCS), and talus medial malleolus space (MCS). CT reconstruction: medial malleolus space of talus (MCS) and inferior tibiofibular space (RFCS). Intraoperative: cotton test, abductor and pronator stress test, lateral forward stress radiograph, anterior drawer test, varus stress radiograph, and ankle radiograph under varus stress. Combined with the imaging signs, trauma history, and physical index examination results of the patients, the diagnosis was made. According to CT reconstruction, X-ray, and intraoperative conditions of each patient and Lauge-Hansen classification, the application value of X-ray and spiral CT three-dimensional reconstruction was analyzed and compared with intraoperative diagnosis as the gold standard.
2. Examination method X-ray film: Philips DR camera was used to perform anteroposterior and lateral X-ray photography for the affected side of the ankle. The CT examination instrument was Toshiba Aquilion 16-Slice Spiral CT Scanner. During the scanning, the patient was placed in supine position. The scanning range was distal to proximal, and the axial scanning range was from 1/3 of the lower tibia to the foot, including the range of 2 cm above and below the fracture line. Parameters: current, 200∼250 mA; voltage, 135 kV; layer thickness, 5 mm; reconstruction spacing, 1 mm; pitch, 1, the standard algorithm for reconstruction calculation. After the scanning, the obtained two-dimensional volume image was transferred to the workstation, and the computer was used to perform three-dimensional image reconstruction, including sagittal and coronal multiplane reconstruction (MPR), maximum density projection (MIP), and surface occlusion imaging (SSD). The free cross-section multiplane recombination mode was used to observe the fracture fragments and details, the surface reconstruction method was used to reconstruct the three-dimensional image of the bone structure around the ankle joint, and the three-dimensional shape of the ankle joint was carefully observed by the maximum density projection.

### 3.1. Observation Indexes and Evaluation Criteria

To compare the diagnosis of different types of ankle fractures by two examination methods. Ankle fractures are classified according to the Lauge–Hansen classification, including pronation-external rotation type (PER), pronation-abduction (PAB), supination external rotation (SER), and supination-adduction (SAB). According to the degree of injury of the patient, the classification of ankle fracture types can be as follows: PER, I∼IV degree; PAB, I∼III degree; SER, I∼IV degree; SAB, I∼II degree.

### 3.2. Statistical Treatment

SPSS 20.0 statistical software was used to process the data. Enumeration data were represented as rate (%), word 2 test was used, measurement data were represented as (*X*- ± *S*), and *P* < 0.05 indicated statistically significant difference [8].

## 4. Results and Discussion

### 4.1. Intraoperative Typing Results

Among the 100 patients, 24 patients were PAB, accounting for 24%, including 12 patients with I degree, 8 patients with critical degree, and 4 patients with radiance. 20 cases belonged to PER, accounting for 20.00%, including 9 cases of I degree, 6 cases of power degree, 3 cases of bulkiness, and 2 cases of compliance; 31 cases (31%) belonged to SAB type, of which 21 cases were I degree and 10 cases were normal degree. 25 cases (25%) were SER, including 13 cases with I degree, 7 cases with power degree, 3 cases with universality degree, and 2 cases with adequacy degree. The diagnostic value of X-ray and spiral CT 3D reconstruction for PAB ankle fracture was found by intraoperative typing results as the gold standard; the specificity, sensitivity, and accuracy of spiral CT 3D reconstruction in the diagnosis of PAB ankle fracture were 100% (91/91), 100% (29/29), and 100% (100/100), respectively, and the X-ray values were 95.6% (87/91), 75.86% (22/29), and 90.83% (109/100), respectively; the specificity, sensitivity, and accuracy of 3D reconstruction of spiral CT were all higher than that of X-ray, and the differences were statistically significant (word 2 = 2.301, 5.849, 11.528; *P* < 0.05), as shown in Table 1.

### 4.2. The Value of X-Ray and Spiral CT 3D Reconstruction in the Diagnosis of PER Ankle Fracture

Using intraoperative typing results as the gold standard, the specificity, sensitivity, and accuracy of spiral CT 3D reconstruction for PER ankle fracture were 100%(96/96), 95.83%(23/24), and 99.17%(119/100), respectively. X-ray values were 93.75% (90/96), 91.67% (22/24), and 93.33% (112/100), respectively; the difference was not statistically significant (word 2 = 0.000; *P*=0.551), and the diagnostic specificity and accuracy of spiral CT 3D reconstruction were both higher than that of X-ray, and the difference was statistically significant (word 2 = 4.301, 4.156; *P* < 0.05), as shown in Table 2.

### 4.3. The Value of X-Ray and Spiral CT 3D Reconstruction in the Diagnosis of SAB Ankle Fracture

Using intraoperative typing results as the gold standard, the specificity, sensitivity, and accuracy of spiral CT 3D reconstruction in the diagnosis of SAB articular fractures were 100% (87/87), 100% (33/33), and 100% (100/100), respectively; X-ray examination was 93.75% (80/87), 91.67% (30/33), and 93.33% (110/100), respectively; there was no significant difference in sensitivity between the two methods (word 2 = 1.397; *P*=0.076). The sensitivity and accuracy of 3D reconstruction of spiral CT were both higher than that of X-ray, and the differences were statistically significant (word 2 = 5.358, 10.435; *P* < 0.05), as shown in Table 3.

### 4.4. Diagnostic Value of X-Ray and Spiral CT 3D Reconstruction in SER Ankle Fracture

Using intraoperative classification as the gold standard, the diagnostic specificity, sensitivity, and accuracy of spiral CT 3D reconstruction for SER ankle fracture were 96.51% (83/86), 97.06% (33/34), and 96.67% (116/100), respectively; X-ray results were 95.35% (82/86), 76.47% (26/34), and 90.00% (108/100), respectively. There was no significant difference in the specificity of the two methods (word 2 = 0.000; *P*=0.670). The sensitivity and accuracy of spiral CT 3D reconstruction diagnosis were higher than that of X-ray. The difference was statistically significant (word 2 = 4.610, 4.286; *P* < 0.05), as shown in Table 4.

## 5. Conclusions

The treatment of ankle fracture is mainly to achieve the best anatomical reduction and fixation, so as to realize the effective recovery of the patient's ankle function. Therefore, strengthening the clinical diagnosis of patients with ankle fracture is of great significance to improve the treatment effect of patients in the future. Ankle fracture is prone to misdiagnosis or missed diagnosis due to its complex anatomical structure, many types of fracture and easy displacement of bone block, which increases the clinical diagnosis difficulty of X-ray and CT scan examination, leading to misdiagnosis or missed diagnosis of ankle fracture. In conclusion, the application of spiral CT reconstruction in the diagnosis of ankle fracture can visually and comprehensively display the fracture site, provide a reliable basis for doctors' clinical diagnosis and treatment, and promote the gradual improvement of patients' clinical treatment effect.

This study retrospectively analyzed the clinical data of patients with ankle fracture admitted to our hospital in the past two years and found that all patients received surgical treatment, preoperative X-ray examination, and spiral CT three-dimensional reconstruction. The intraoperative typing results showed that, of the 100 patients, 20 (20.00%) were found to have pronation and extrapolation (PER), 24 (24%) to have pronation and extrapolation (SER), and 25 (25%) to have pronation and adduction (SAB), respectively. Using the intraoperative classification results as the gold standard, the diagnostic accuracy of spiral CT 3D reconstruction for different types of ankle fracture was higher than that of X-ray, suggesting that the application of spiral CT 3D reconstruction in the early diagnosis of different types of ankle fracture has more clinical application value than that of X-ray. In conclusion, the application of spiral CT three-dimensional reconstruction in the early diagnosis of ankle fracture can accurately detect the classification of patients, which has important clinical application value and can be used as the first choice for the early classification diagnosis of ankle fracture.

## Figures and Tables

**Table 1:** Comparison of the value of X-ray and spiral CT 3D reconstruction in the diagnosis of PAB type of ankle fracture.

X-ray	Intraoperative		A combined	CT	Intraoperative		A combined
	+	−			+	−	
+	20	3	23	+	25	0	25
−	7	70	77	−	0	75	75
A combined	27	73	100	A combined	25	75	100

**Table 2:** Comparison of diagnostic value of 2X scan and spiral CT 3D reconstruction in PER ankle fracture.

X-ray	Intraoperative		A combined	CT	Intraoperative		A combined
	+	−			+	−	
+	18	3	21	+	19	0	19
−	1	78	79	−	1	80	81
A combined	19	81	100	A combined	20	80	100

**Table 3:** Comparison of X-ray and spiral CT 3D reconstruction in the diagnosis of SAB ankle fracture.

X-ray	Intraoperative		A combined	CT	Intraoperative		A combined
	+	−			+	−	
+	22	5	27	+	31	0	31
−	1	72	73	−	0	69	69
A combined	23	77	100	A combined	31	69	100

**Table 4:** Comparison of the diagnostic value of X-ray and spiral CT 3D reconstruction in SER ankle fracture.

X-ray	Intraoperative		A combined	CT	Intraoperative		A combined
	+	−			+	−	
+	16	4	20	+	17	7	24
−	5	75	80	−	1	75	76
A combined	21	79	100	A combined	18	82	100

## Data Availability

The data used to support the findings of this study are available from the corresponding author upon request.
